The article "A Novel Fault Diagnosis Method for Denoising Autoencoder Assisted by Digital Twin" was published in 2022. Journal: Comput Intell Neurosci.

# A Novel Fault Diagnosis Method for Denoising Autoencoder Assisted by Digital Twin

**DOI:** 10.1155/2022/5077134

**Published:** 2022-07-21

**Authors:** Wenan Cai, Qianqian Zhang, Jie Cui

**Affiliations:** ^1^School of Mechanical Engineering, Jinzhong University, Jinzhong 030619, China; ^2^School of Automation and Software Engineering, Shanxi University, Taiyuan 030006, China; ^3^School of Mechanical Engineering, North University of China, Taiyuan, Shanxi 030051, China

## Abstract

Digital twin (DT) is an important method to realize intelligent manufacturing. Traditional data-based fault diagnosis methods such as fractional-order fault feature extraction methods require sufficient data to train a diagnosis model, which is unrealistic in a dynamically changing production process. The ultrahigh-fidelity DT model can generate fault state data similar to the actual system, providing a new paradigm for fault diagnosis. This paper proposes a novel digital twin-assisted fault diagnosis method for denoising autoencoder. First, in order to solve the problem of limited or unavailable fault state data for machines in dynamically variable production scenarios, a DT model of the machine is established. The model can simulate a dynamically changing production process, thereby generating data for different failure states. Second, a novel denoising autoencoder (NDAE) with Mish as the activation function is proposed and trained using the source domain data generated by DT. Finally, in order to verify the effectiveness and feasibility of the proposed method, the method is applied to a fault diagnosis example of a triplex pump, and the results show that the method can realize intelligent fault diagnosis when the fault state data are limited or unavailable.

## 1. Introduction

As intelligent manufacturing becomes increasingly automated, digitized, and intelligent, more attention is paid to manufacturing process reliability and safety [1–3]. Minor failures in the production process can cause irreparable damage. Therefore, fault diagnosis is an important aspect of intelligent manufacturing [4–6]. Among the current machine learning methods, support vector machines, decision trees, and fractional order have been successfully applied in the field of fault diagnosis [7, 8]. In recent years, deep learning methods such as Bayesian networks, long short-term memory, and convolutional neural networks have been very popular in fault diagnosis due to their powerful modeling and representation capabilities [9–12]. The methods mentioned above can significantly improve the accuracy and efficiency of fault diagnosis under certain conditions. However, in order to obtain high fault diagnosis accuracy for deep learning methods, the primary condition is that the source domain data should be sufficient and contain comprehensive fault diagnosis information. In practical industrial applications, machines are often in a dynamically changing production environment, and the health and fault information collected at this time are uncertain. Therefore, in the dynamically changing production process, it is difficult to collect a large amount of labeled fault data [13]. In addition, the machine is time-consuming and laborious to complete the degradation process, and the cost of marking a large amount of fault data is high. In order to prevent catastrophic accidents, many enterprises and factories do not allow machines to run to failure. Therefore, the above intelligent fault diagnosis methods are difficult to play a role in the dynamic changing production process [14].

The article "A Novel Fault Diagnosis Method for Denoising Autoencoder Assisted by Digital Twin" was published in 2022. Journal: Comput Intell Neurosci.

In order to solve the above problems of insufficient training data and incomplete diagnostic information, some scholars have thought of transfer learning methods. This method can transfer a large amount of diagnostic information collected on a specific experimental platform to dynamically changing production scenarios, solving the problem of insufficient training data [15]. For example, Zhang et al. proposed a first-layer wide convolutional deep neural network (WDCNN), the key of which is to use large convolution kernels in the first layer of convolution to extract short-term features. The convolution kernel parameters of the remaining convolutional layers except the first layer are reduced, which is conducive to deepening the network and suppressing overfitting [16]. Zhang et al. proposed a new CNN model, the advantage of which is that it does not require signal denoising preprocessing, which can realize fault diagnosis in noisy environments and variable working conditions [17]. Ren et al. proposed a new fault detection and classification method (DRCNN), which designed an important module “multiscale summation” for deep feature extraction. This method can combine features of multiple scales and different levels from unequal layers, which ensures the completeness of information [18]. However, the robustness of the diagnostic performance of transfer learning suffers in scenarios where working conditions and system characteristics are not fixed. Parameter transfer learning methods can assume that some parameters are shared between source tasks and target tasks, or the prior distribution of model hyperparameters is shared. Then, we use a small number of samples in the target domain to fine-tune the pretrained model, improve the overall performance of the model, and achieve a more robust fault diagnosis effect. However, the parameter transfer learning method also faces the problem of incomplete diagnostic information in the source domain [19].

The article "A Novel Fault Diagnosis Method for Denoising Autoencoder Assisted by Digital Twin" was published in 2022. Journal: Comput Intell Neurosci.

With the rapid development and application of information technology, in recent years, digital twin (DT) technology has received more and more attention in various fields, such as product design and manufacturing, medical analysis, engineering construction, process optimization, and job shop scheduling. [20–22]. Also in the field of intelligent manufacturing, DT technology has also played a pivotal role and has become a powerful weapon to promote the development of intelligent manufacturing. It makes full use of physical model, sensor update, operation history, and other data, integrates multidisciplinary, multiphysical, multiscale, multiprobability simulation process, and completes the mapping in virtual space, thereby reflecting the full life cycle process of the corresponding physical equipment. DT technology can not only reduce design and maintenance costs but also improve manufacturing efficiency and quality. Ultrahigh-fidelity DT models can generate simulated data close to real systems, providing new opportunities for intelligent fault diagnosis. Wang et al. proposed a DT reference model for rotor system fault diagnosis. The requirements for building a digital twin model are discussed, and a model update scheme based on parameter sensitivity analysis is proposed to improve the adaptability of the model [23]. Jain et al. constructed a digital twin that can estimate the measurable characteristic output of a photovoltaic energy conversion unit (PVECU) in real time. A PVECU consists of a photovoltaic source and a source-level power converter [24]. Qin et al. proposed a full life cycle rolling bearing DT model driven by a combination of data and models. Through an improved CycleGAN neural network, the simulated data in the virtual space are mapped to the physical space, and the results of the DT model are compared with the measured signals in the time and frequency domains to verify the effectiveness and feasibility of the proposed model [25]. Xu et al. proposed a two-stage DT fault diagnosis method (DFDD) based on deep transfer learning, which realizes fault diagnosis in the development and maintenance stages [26]. Qin et al. proposed a digital twin convolutional neural network model with multidomain input (DTCNNMI) in order to realize the misfire diagnosis of the diesel engine in a strong noise environment and different operating conditions [27]. However, most of the current research focuses on the conceptual model and key technologies of DT, and few people conduct more specific research on the fault diagnosis framework, mechanism, and algorithm to overcome the practical problem of limited diagnostic data.

The article "A Novel Fault Diagnosis Method for Denoising Autoencoder Assisted by Digital Twin" was published in 2022. Journal: Comput Intell Neurosci.

In this paper, a novel digital twin-assisted fault diagnosis method for denoising autoencoder is proposed for the problem of machine intelligence fault diagnosis. The DT model can simulate a dynamically changing production process, thereby generating data of different fault states, and solving the problem of limited or unavailable fault state data for machines under dynamically variable production conditions. The main contributions of this paper are as follows:

1. A DT-assisted deep transfer learning fault diagnosis method is proposed, which is mainly used for fault diagnosis experiments of triplex pumps. A DT model of the machine is established to simulate the dynamically changing production process, thereby generating data for different failure states. The DT model is continuously updated during this process. The method solves the problem that the fault state data are limited or not used when the working state of the machine changes and the system characteristic changes.
2. A novel denoising autoencoder (NDAE) with Mish as the activation function is proposed, which has the properties of no upper bound, lower bound, smoothness, and nonmonotonicity compared with other activation functions.
3. A sparse penalty term is introduced to fully combine the advantages of sparse autoencoders and denoising autoencoders to effectively learn sparse feature representations from noisy samples.

## 2. Theoretical Background of Autoencoders

Convolutional neural network (CNN) is a commonly used network structure in deep learning methods and is currently widely used in the field of intelligent fault diagnosis of mechanical systems. However, the structure of CNN is relatively complex, and the amount of computation is relatively large compared with other deep learning methods. Compared with CNN, autoencoder has a simpler structure and stronger operability, which can train the model more easily and effectively. A type of neural network, after training, attempts to copy the input to the output. At present, many improved forms have been derived from the autoencoder. On the basis of the autoencoder, the noise reduction autoencoder adds noise to the input data of the input layer in order to prevent the overfitting problem, so that the learned encoder is more robust. A sparse autoencoder is a special three-layer neural network with sparse constraints added to the general neural network. From the input layer to the hidden layer, the high-dimensional data are mapped to the low-dimensional data, and the projected low-dimensional data are restored to the original high-dimensional data from the hidden layer to the output layer [28]. Assuming that *x*=[*x*_1_, *x*_2_, ..., *x*_*m*_] is a labeled m-dimensional real sample, the formula for noise sample $\tilde{x}=\left[\tilde{x_{1}},\tilde{x_{2}},...,{\tilde{x}}_{m}\right]$ is defined as follows:

(1) $$\begin{array}{c} \tilde{x}=x+N\left(0,\delta^{2}Ι\right), \end{array}$$

where *N*(0, *δ*^2^Ι) represents Gaussian noise with noise level *δ*.

The article "A Novel Fault Diagnosis Method for Denoising Autoencoder Assisted by Digital Twin" was published in 2022. Journal: Comput Intell Neurosci.

Then, the formulas of the feature vectors $\tilde{h}=\left[{\tilde{h}}_{1},{\tilde{h}}_{2},...,{\tilde{h}}_{n}\right]$ and reconstruction vectors $\tilde{z}=\left[{\tilde{z}}_{1},{\tilde{z}}_{2},...,{\tilde{z}}_{m}\right]$ of the noise samples are as follows:

(2) $$\begin{array}{c} \tilde{h}=f_{H}\left(w^{\left(1\right)}\tilde{x}+b^{\left(1\right)}\right),\\ \tilde{z}=f_{O}\left(w^{\left(2\right)}\tilde{h}+b^{\left(2\right)}\right), \end{array}$$

where *f*_*H*_ and *f*_*O*_ are the activation functions of the hidden layer and the output layer. (**w**^(1)^,**b**^(1)^) is the weights and biases of the input and hidden layers. Similarly, (**w**^(2)^,**b**^(2)^) is the weight and bias of the hidden layer and the output layer.

The formulas of the loss function *l*_1_, sparse penalty term *l*_2_, and weight decay term *l*_3_ of MSE are expressed as follows:

(3) $$\begin{array}{c} l_{1}=\frac{1}{2}\sum_{i=1}^{m}{\left({\tilde{z}}_{i}-x_{i}\right)}^{2},\\ l_{2}=\beta \left(\sum_{j=1}^{n}r\;\log\frac{r}{{\hat{r}}_{j}}+\left(1-r\right)\log\frac{1-r}{1-{\hat{r}}_{j}}\right),\\ l_{3}=\frac{\lambda }{2}\left(\sum_{i=1}^{m}\sum_{j=1}^{n}\left({\left(w_{ji}^{\left(1\right)}\right)}^{2}+{\left(w_{ji}^{\left(2\right)}\right)}^{2}\right)\right), \end{array}$$

where *β* is the sparse penalty factor. *r* is the sparse constant. *λ* is the weight decay factor. *w*_*ji*_^(1)^ is the connection weight between the *i*th input unit and the *j*th hidden unit. Similarly, *w*_*ji*_^(2)^ is the connection between the *j*th hidden unit and the *i*th output unit connection weight.

Then, the overall loss function can be expressed as follows:

(4) $$\begin{array}{c} \left(L_{S}=l_{1}+l_{2}+l_{3}\right). \end{array}$$

## 3. Proposed Method

### 3.1. NDAE Method

The NDAE method proposed in this paper is inspired by reference [28]. Based on the combination of sparse autoencoder and denoising autoencoder into sparse denoising autoencoder, a sparse penalty term is introduced, which can effectively learn the sparse features of noise samples. In addition, inspired by reference [29], the Mish activation function with stronger learning ability is adopted. The ReLU activation function is the most widely used activation function in neural networks, and it mainly has the characteristics of having no upper bound and having a lower bound, which greatly limits its learning ability. Compared with ReLU, the Mish activation function has the characteristics of smoothness and nonmonotonicity. The smooth characteristics can make the network easier to optimize and improve the generalization performance, and the nonmonotonicity characteristics can improve the interpretability of the network. Comparison results on several datasets verify that Mish's metrics outperform ReLU and other activation functions for most tasks [29]. The waveform of the Mish function is shown in Figure 1. It can be seen from the figure that it allows a small negative gradient to flow in when it is negative, thereby ensuring information transfer and eliminating the dying ReLU phenomenon. The mathematical expression of the Mish activation function is as follows:

(5) $$\begin{array}{c} f_{M}\left(x\right)=x\;\tanh\left(\text{softplus}\left(x\right)\right)\\ =x\;\tanh\left(ln\left(1+e^{x}\right)\right),\\ \tanh\left(x\right)=\frac{\left(e^{x}-e^{-x}\right)}{\left(e^{x}+e^{-x}\right)},\\ \text{softplus}\left(x\right)=\log\left(1+e^{x}\right). \end{array}$$

Mish is unbounded above and bounded below, and its first derivative can be defined as follows:

(6) $$\begin{array}{c} f^{\prime }\left(x\right)=\frac{e^{x}\omega }{\delta^{2}}, \end{array}$$

where (*ω*=4(*x*+1)+4*e*^2*x*^+*e*^3*x*^+*e*^*x*^(4*x*+6)), (*δ*=2*e*^*x*^+*e*^2*x*^+2).

The article "A Novel Fault Diagnosis Method for Denoising Autoencoder Assisted by Digital Twin" was published in 2022. Journal: Comput Intell Neurosci.

The Mish activation function adds smoothness and nonmonotonicity to the ReLU activation function. These features can effectively retain the negative information of the data, make up for the deficiencies of ReLU, help information transfer, and have better expressiveness. It can be seen from formula (6) that the first derivative of the Mish activation function is differentiable; that is, the Mish activation function is continuously differentiable. This feature avoids singularities and thus avoids unwanted side effects when performing gradient-based optimization problems using the Mish activation function. In order to make the reconstructed output of the NDAE method infinitely close to the original input, a sigmoid activation function is selected at the output layer to normalize the input to the range of [0, 1] into account. So the hidden and reconstructed outputs using the Mish activation function are

(7) $$\begin{array}{c} \tilde{h}=f_{M}\left(w^{\left(1\right)}\tilde{x}+b^{\left(1\right)}\right),\\ \tilde{z}=f_{S}\left(w^{\left(2\right)}\tilde{h}+b^{\left(2\right)}\right), \end{array}$$

where *f*_*M*_ and *f*_*S*_ are the Mish and sigmoid activation functions, respectively.

To ensure that the real samples and the samples generated by the NDAE reconstruction are as similar as possible, the difference between the real samples and the reconstructed samples is reduced. To further measure the local similarity between the two, use the maximum correlation entropy instead of MSE, and use the gradient descent algorithm to adjust **w** and **b**, the correlation formula is as follows:

(8) $$\begin{array}{c} w_{q+1}=w_{q}-\xi_{q}\left(\frac{\partial L_{N}}{w_{q}}\right)+\varepsilon \left(w_{q}-w_{q-1}\right),\\ b_{q+1}=b_{q}-\xi_{q}\left(\frac{\partial L_{N}}{b_{q}}\right)+\varepsilon \left(b_{q}-b_{q-1}\right), \end{array}$$

where *q* is the current number of iterations. *L*_*N*_ is the total loss function of the proposed method NDAE. *ξ*_*q*_ is the current learning rate. *ε* is the momentum factor. Then, the NDAE total loss function is as follows:

(9) $$\begin{array}{c} \left(L_{N}=-l_{4}+l_{2}+l_{3}\right), \end{array}$$

where *l*_4_ is the formula of maximum correlation entropy, which is more effective in local similarity measurement of complex signals than MSE. The formula for *l*_4_ is as follows:

(10) $$\begin{array}{c} l_{4}=\frac{1}{\sqrt{2\pi }\tau }\sum_{i=1}^{m}\exp\left(-\frac{{\left(\tilde{z_{i}}-x_{i}\right)}^{2}}{2\tau^{2}}\right),\\ \xi_{q+1}=\frac{\xi_{q}}{\rho }, \end{array}$$

where *τ* is the kernel width adjustment parameter. *ρ* is the decay factor. Using multiple NDAEs with softmax classifiers can be constructed to stack NDAEs to improve learning ability.

The article "A Novel Fault Diagnosis Method for Denoising Autoencoder Assisted by Digital Twin" was published in 2022. Journal: Comput Intell Neurosci.

### 3.2. DT-Assisted NDAE Method

To solve the problem of limited or unavailable fault state data for machines under dynamically variable production conditions, a DT-assisted NDAE method is proposed in this paper. The overall framework of the method is shown in Figure 2. The green part is the construction part of the DT model of the triplex pump. First, the simulation model of the real machine needs to be established, and then, the simulation model needs to be continuously updated to adapt to the dynamic and variable production environment. This paper updates the simulation model by minimizing the difference in system response between the simulation model and the measured data. The adaptively updated DT model is then used to simulate the fault state of the machine, generating comprehensive fault data required for fault diagnosis. The blue part in Figure 2 is the parameter transfer learning part of the new denoising autoencoder. First, the stacked NDAE model is constructed using the Mish activation function and maximum correlation entropy in 3.1, and then, a large amount of fault state data generated by the DT model are used as the training data in the source domain, which is input into the stacked NDAE model for pretraining. Finally, parameter transfer learning can greatly improve the training efficiency of stacked NDAE, so the parameter transfer learning method is used to realize machine fault diagnosis. It is worth noting that this paper selects a sample in the target domain to fine-tune the pretrained stacked NDAE to further adjust the model parameters.

The article "A Novel Fault Diagnosis Method for Denoising Autoencoder Assisted by Digital Twin" was published in 2022. Journal: Comput Intell Neurosci.

The shared parameters for parameter transfer learning in this paper are all hyperparameters, weights, and biases. It is worth noting that all weights and biases are pretrained before fine-tuning to ensure the effectiveness of parameter transfer learning.

## 4. Case Analysis

### 4.1. Experimental Description

In order to evaluate the effectiveness and feasibility of the proposed method, the method is applied to a fault diagnosis example of a triplex pump. The DT model of the triplex pump is shown in Figure 3. Inspired by reference [30], this paper imitates reference [30] and uses the Simscape module in Matlab to create a simulation model of a triplex pump. Triplex pumps have a crankshaft driving three plungers. Compared to single-piston pumps, one air chamber of the plunger is always vented, resulting in smoother flow and less pressure variation, thereby reducing material strain. The parameter values were then automatically tuned using Simulink design optimization so that the model produced results that matched the measured data to simulate the system behavior of a triplex pump in a dynamically variable production environment. Simulink design optimization selects parameter values for simulation, calculates the difference between the simulation curve and the measured curve to update the simulation model, and generates a simulation model with the system response function of modifying model parameters. Based on this difference, new parameter values are selected for a new simulation. The gradient of the parameter value is calculated to determine the direction in which the parameter should be adjusted. The DT model update of the triplex pump in this study is implemented through Simulink design optimization and automatically tunes the parameter values so that the model generates results that match the measured data.

The DT model of the triplex pump can simulate three typical pump failures, including seal leakage from the plunger, inlet blockage, and increased friction due to bearing wear. These fault conditions can be configured and toggled through the pump module dialog or commands. This paper collects data for seven fault states, including healthy state, three single faults, and three composite faults. Dataset A and dataset B are collected by simulating two scenarios. Dataset A is simulation data with original parameters. Dataset B is simulation data collected when working conditions and system characteristics change, that is, actual situation data.  Table 1 shows the detailed description of dataset A and dataset B, 125 samples are selected for each fault state, and each sample contains 1200 data points.  Table 2 shows the detailed settings of the DT-assisted NDAE parameter transfer learning task.  Table 3 shows the hyperparameter settings for stacked NDAE. The size of the first, second, and third hidden layers and other network structures are determined by experiments and experience. The number of iterations, initial learning rate, decay factor, and momentum are determined empirically, respectively. The selection of other hyperparameters is mainly based on reference [25].

The article "A Novel Fault Diagnosis Method for Denoising Autoencoder Assisted by Digital Twin" was published in 2022. Journal: Comput Intell Neurosci.

### 4.2. Comparison Method

To verify the effectiveness and feasibility of the proposed method, it is compared with several state-of-the-art methods. Both the comparison method and the proposed method are tested using the fault data generated by the DT model.

1. SVM. The SVM algorithm is used to realize the fault classification of the triplex pump. SVM is a binary classification model that maps feature vectors to points in space, and its purpose is to find a line to better distinguish these points. Before the advent of deep learning, SVM was considered to be the better-performing algorithm in machine learning.
2. Stacked SDAE method. Stacked denoising autoencoders with ReLU as activation function.
3. LeNet-5 CNN. Fault classification of triplex pumps using a classic LeNet-5 convolutional neural network.

### 4.3. Experimental Results and Analysis

In this experiment, the effectiveness and feasibility of the proposed NDAE method are verified by the parameter transfer learning method. First, 75 samples are randomly selected from the 125 samples of dataset A as training samples in the source domain, and these 75 samples are input into the NDAE network for pretraining. Then, one sample is used from dataset B to fine-tune the pretrained network. This is because the DT model of the triplex pump can generate the data of the fault state,so just select a sample from the target domain to fine-tune the pretrained stacked NADE, and further construct the deep structure NADE to obtain better fault diagnosis results. Finally, 50 samples are used from dataset B for testing. In order to reduce the influence of random factors, the experiments were repeated six times; that is, six independent experiments were carried out using random samples for each method. The fault diagnosis accuracy of six experiments is shown in Figure 4. It can be seen from Figure 4 that the diagnostic accuracy of the six experiments exceeds 90%, and the average fault diagnosis accuracy is 92.4%.

The article "A Novel Fault Diagnosis Method for Denoising Autoencoder Assisted by Digital Twin" was published in 2022. Journal: Comput Intell Neurosci.

To verify the effectiveness and feasibility of the proposed method, it is compared with SVM, stacked SDAE method, and LeNet-5 CNN method. To reduce the influence of random factors, the experiments were repeated six times; that is, six independent experiments were performed using random samples for each method. The experimental results are shown in Figure 5. The average accuracy of the SVM method, stacked SDAE method, and LENet-5 CNN method is 76.5%, 87.8%, and 88.6%, respectively. It can be seen from the experimental results that the proposed method has higher fault diagnosis accuracy and is more conducive to the fault classification of the triplex pump.

## 5. Conclusion

In this paper, a DT-assisted NDAE parameter transfer learning fault diagnosis method is proposed, which is mainly used in the fault diagnosis experiment of the triplex pump. This method is designed to achieve high-accuracy fault classification when measurement data are insufficient or unavailable. We use the digital twin model of the machine to generate fault state data similar to the actual system to make up for the lack of data. In addition, the stacked autoencoder is improved, and the Mish activation function has no upper bound, lower bound, nonmonotonicity, and smoothness to increase the generalization performance of the network and the interpretability of the network. This ensures information transfer and eliminates the dying ReLU phenomenon. Finally, by generating simulation data of the triplex pump under various fault conditions, the effectiveness of fault diagnosis of the proposed NDAE method is verified. The results show that the ultrahigh-fidelity DT model can generate simulated data close to the real system, providing new opportunities for intelligent fault diagnosis. The DT-assisted NDAE parameter transfer learning fault diagnosis method can realize intelligent fault diagnosis of mechanical systems in dynamically changing production environments.

Although the DT-assisted NDAE parameter transfer learning fault diagnosis method can effectively improve the fault diagnosis accuracy of the model, the construction of the machine's DT model is a difficulty of this method. Therefore, the following research focuses on making full use of the main mechanism of DT to build DT models of other basic components such as bearings and combining deep transfer learning methods to improve fault diagnosis performance. How to further combine DT and deep transfer learning is the focus and difficulty of the next research.

## Figures and Tables

**Figure 1:** Mish activation function waveform.

**Figure 2:** General framework of DT-assisted deep transfer learning method.

The article "A Novel Fault Diagnosis Method for Denoising Autoencoder Assisted by Digital Twin" was published in 2022. Journal: Comput Intell Neurosci.

**Figure 3:** DT model of triplex pump.

**Figure 4:** The fault diagnosis accuracy of the proposed method in ten experiments.

**Figure 5:** Fault diagnosis accuracy of four methods.

**Table 1:** Seven working states of triplex pump.

Datasets	Working status	Number of samples	Labels
A/B	Healthy	125	1
	Seal leak	125	2
	Blocked inlet	125	3
	Bearing wear	125	4
	Seal leak and blocked inlet	125	5
	Seal leak and bearing wear	125	6
	Blocked inlet and bearing wear	125	7

**Table 2:** Detailed settings of parameter transfer tasks.

Method	Source domain training/test samples	Number of training/testing samples
Parameter transfer learning	Dataset A/B	75/50

**Table 3:** Hyperparameter settings for stacked NDAE methods.

Hyperparameters	Value	Hyperparameters	Value
The size of the first hidden layer	450	Kernel width	1.2
The size of the third hidden layer	100	Sparse penalty factor	5
Number of iterations	60	Initial learning rate	0.01
Weight decay coefficient	0.004	Decay factor	1.1
Noise level	0.08	Momentum	0.8

## Data Availability

No new data were created or analyzed in this study. Data sharing is not applicable to this article.
